# The Value of Nuclear Magnetic Resonance in Liver Nodular Lesions

This article has been retracted.

**DOI:** 10.1155/2022/8165950

**Published:** 2022-08-11

**Authors:** Si Chen, JiaLing Bao

**Affiliations:** Wuxi Second People's Hospital, Wuxi 214000, Jiangsu, China

## Abstract

In order to analyze the value of contrast-enhanced ultrasound (CEUS) combined with functional magnetic resonance imaging (fMRI) in the early differential diagnosis of liver nodular lesions, the authors studied the value of MRI in liver nodular lesions. A total of 82 patients with liver nodular lesions admitted to the hospital were selected for retrospective analysis; all of them underwent CEUS and fMRI examinations, and taking a biopsy or postoperative pathological examination results as the gold standard, the diagnostic value of CEUS, fMRI single item, and the two combined examinations for liver nodular lesions was analyzed by four-table. The biopsy or postoperative pathological examination results showed that a total of 88 lesions were detected in 82 patients, including 51 patients with benign lesions, with 54 lesions, and 31 patients with malignant lesions, with 34 lesions. Taking biopsy or pathological examination results as the gold standard, the four-table analysis CEUS had a sensitivity of 79.63%, a specificity of 82.35%, an accuracy of 80.68%, and a Kappa value of 0.603 for diagnosing benign and malignant liver nodular lesions. The sensitivity of fMRI in diagnosing benign and malignant liver nodular lesions was 83.33%, the specificity was 85.29%, the accuracy was 84.09%, and the Kappa value was 0.672; the combined sensitivity of the two in the diagnosis of benign and malignant liver nodular lesions was 94.44%, the specificity was 91.18%, the accuracy was 93.18%, and the Kappa value was 0.856, both of which were superior to single detection, and the difference in accuracy was statistically significant (*χ*^2^  = 5.683, *P* < 0.05). CEUS and fMRI have a certain value in the differential diagnosis of liver nodular lesions; the combination of the two can improve the diagnostic sensitivity and accuracy, and has more clinical application value.

## 1. Introduction

Among the nodular lesions of the liver, the incidence of benign nodular lesions is significantly higher than that of malignant lesions, including hepatic cysts, hepatic cavernous hemangioma, focal nodular hyperplasia, hepatic adenoma, and inflammatory lesions. In recent years, the wide application of multi-slice spiral CT (MSCT), magnetic resonance imaging (MRI), ultrasound, positron emission computed tomography (PET or PET-CT) and other technologies have contributed to the accurate and specific detection of liver lesions. Diagnosis provides support [1]. Some lesions can be assessed at the molecular level, which is conducive to accurate diagnosis of lesions before treatment. With its excellent soft tissue resolution, no radiation damage, and the advantages of any direction and multi-parameter imaging, MRI can reflect the morphology, signal characteristics, and tissue biochemical components of liver nodular lesions from various aspects, as shown in Figure 1; Dynamic contrast-enhanced MRI, perfusion imaging, and MR angiography (MRA) can show the hemodynamic changes and vascular morphology of nodular lesions; MR cholangiopancreatography (MR cholopancreatography, MRCP) is the use of water imaging technology to display the situation of intrahepatic and extrahepatic bile ducts [2]. At present, MRI is more and more widely used in the diagnosis of liver lesions, and the efficiency of imaging diagnosis is equal to or slightly higher than that of MSCT. The new progress of MRI in recent years is mainly manifested in two aspects: the application of tissue-specific contrast agents and the development of scanning sequences. The application of a number of new scanning sequences of magnetic resonance makes it possible to perform functional imaging and molecular imaging of the liver [3]. Diffusion-weighted imaging (DWI) is currently the most widely used, which can be used for preliminary characterization by detecting the movement of water molecules and the apparent diffusion coefficient (ADC value) to reflect the characteristics of lesions, and background suppression diffusion-weighted imaging (DWIBS), the application is conducive to the sensitive detection of large-scale and even systemic lesions and improves the disease diagnosis rate.

## 2. Literature Review

Citone et al. found that Gd-EOB-DTPA was able to delineate liver enhancement abnormalities in young patients soon after Fontan surgery, suggesting that this noninvasive technique may be a useful method to detect early FALD. Gd-EOB-DTPA MRI before treatment can predict efficacy, and patients with stronger delayed enhancement respond better to treatment and live longer [4]. Chilamkurti et al investigated the clinical feasibility of preoperative routine clinical dynamic Gd-EOB-DTPA-enhanced MRI alone in predicting posthepatectomy liver failure (PHLF) in patients with HCC. The results indicated that residual liver function parameters estimated preoperatively according to the routine clinical dynamic Gd-EOB-DTPA-enhanced MRI protocol could predict postoperative liver failure in HCC patients, and may be better than conventional methods [5]. Vernuccio et al found that Gd-EOB-DTPA-enhanced MRI can improve the differential diagnosis of liver cancer and FNH [1]. Ajay et al found that the application of Gd-EOB-DTPA-enhanced hepatobiliary specific phase scan can improve the differential diagnosis of benign and malignant liver lesions [6]. Liu et al. A study comparing the diagnostic accuracy of contrast-enhanced ultrasonography and Gd-EOB-DTPA-enhanced MRI scans for focal liver lesions in patients with cirrhosis showed that the sensitivity and specificity of contrast-enhanced ultrasonography in diagnosing liver cancer were 92% and 50.0%, respectively; the sensitivity and specificity of Gd-EOB-DTPA-enhanced MRI were 90.2% and 83.3%, respectively [7]. Zhang et al. evaluated EUS-guided fine needle aspiration (FNA) as a diagnostic method for focal liver lesions, although it has a high diagnostic yield, the safety and cost-effectiveness of this procedure still need to be further explored [8]. Snast et al. are investigating the diagnostic value of CEUS and sulfur hexafluoride (SF) with MRI and liver-specific contrast agent Gd-EOB-DTPA for hepatocellular adenoma and FNH. The results showed that CEUS and MRI appearances of liver-specific contrast agents were fairly consistent in the diagnosis of HCA and FNH. The diagnostic accuracy of MRI with liver-specific contrast agents is significantly higher than that of CEUS [9]. Wu et al. reported an association between RE representing hepatic uptake of Gd-EOB-DTPA and the METAVIR scoring system used to differentiate normal liver parenchyma from higher stages of hepatic fibrosis [10]. Bai et al demonstrate that high intensity on DWI, coupled with high signal intensity on T2, is the most specific feature to distinguish atypical HCC from dysplastic nodules (sensitivity 80.0%, specificity 100%, positive predictive value 100%, and negative predictive value 78.3%). In most cases, gadolinic acid improves the detection of focal liver lesions and can be classified from LGDN, HGDN, and early HCC lesions, thereby avoiding liver biopsy [11]. In the past, the diagnosis of liver nodular lesions mostly relied on enhanced X-ray computed tomography (CT), contrast-enhanced ultrasound (CEUS) is more safe, simple, painless, and has clearer images, and functional magnetic resonance imaging (fMRI) has the advantages of noninvasiveness and no radiation exposure. Studies have reported that both of them have certain diagnostic value for liver nodular lesions, and are highly accepted by patients, but it is difficult to characterize the nature of the disease with a single detection method. At present, there are few studies on the differential diagnosis value of the combined examination of the two in liver nodular lesions. Therefore, this study intends to explore the CEUS combined with fMRI in the diagnosis of early liver nodular lesions, in order to provide a certain reference value for clinical application.

## 3. Research Methods

### 3.1. General Information

From March 2018 to December 2021, 82 patients with liver nodules who were admitted to a maternal and child health hospital and a cancer hospital in a certain place were selected for retrospective analysis, including 43 males and 39 females; Aged 28–79 years, with an average age (52.49 ± 12.16) years old. Among the 82 patients with liver nodules, 5 had hepatitis B, 32 had abdominal discomfort, abdominal distension, abdominal pain, and other symptoms, and 28 had elevated alanine aminotransferase and aspartate aminotransferase, and 14 had elevated alpha-fetoprotein levels, 3 cases of mild jaundice. All patients underwent CEUS and fMRI examinations, which were confirmed by biopsy or postoperative pathological examination [12].

### 3.2. Inclusion and Exclusion Criteria

1. Inclusion criteria are as follows: (1) Clinical diagnosis of liver nodules based on typical imaging findings; (2) Complete clinical data; (3) Signed informed consent.
2. Exclusion criteria are as follows: (1) Have a history of surgical resection; (2) Women who are pregnant or breastfeeding; (3) Those who are allergic to Sonovit; (4) The compliance is not high and cannot cooperate with the researcher.

### 3.3. Instruments and Reagents

Sequoia 512 color Doppler diagnostic instrument; 1.5 T HDx magnetic resonance scanner; Sonovel contrast agent.

### 3.4. Inspection Method

#### 3.4.1. CEUS Inspection

Patients were fasted before the examination to reduce intestinal gas interference. Using color Doppler diagnostic equipment, 4c contrast probe, frequency 2∼4 MHz. Intravenous injection of sonovir contrast agent (2.4 ml), the patient was placed in the supine position and the lateral position, and the right subcostal margin and the right intercostal space were obliquely scanned, respectively, and the right subcostal margin, the right rib, and the right intercostal region were scanned longitudinally. The upper abdomen was swept under the sword, and the location, size, shape, boundary, and internal echo characteristics of the nodular lesions were recorded. Angiographic images were recorded, arterial (15–30 s), portal phase (31–120 s), and delayed phase (121–360 s).

#### 3.4.2. fMRI examination

The fMRI examination was performed using a magnetic resonance scanner and an 8-channel phased array body coil. The scanning range is from the top of the diaphragm to the lower border of the liver. Conventional sequence T_1_-weighted imaging (T1WI), T_2_-weighted imaging (T_2_WI), diffusion-weighted imaging (DWI), T_2_WI, and susceptibility-weighted imaging (susceptibility-weighted imaging, SWI) scan.

### 3.5. Observation and Evaluation Indicators

The location, size, shape, boundary, and enhancement of the nodular lesions in the liver were observed and recorded [13]. CEUS and fMRI examinations were performed on the patients by 2 senior radiologists using a double-blind method, and the results were the same as the final examination results, if there is any objection, a third senior physician will be introduced, and the final result will be decided through consultation.

### 3.6. Statistical Methods

SPSS25.0 software was used for statistical analysis of the data, and the count data was expressed as [case (%)], and the comparison was made by X^2^ test or Fisher's exact probability method; Taking biopsy or postoperative pathological examination results as the gold standard, the diagnostic value of CEUS and fMRI examinations for liver nodular lesions was evaluated by a four-table. Table and the consistency test (Kappa test) were performed. *P* < 0.05  was considered to be statistically significant.

The mathematical definition formula for the correlation analysis of factors using the X^2^ test is shown in the following formula:

(1) $$\begin{array}{c} \chi^{2}=\sum_{i=1}^{r}\overset{c}{\underset{j=1}{\sum }}\frac{{\left(f_{ij}^{0}-f_{ij}^{e}\right)}^{2}}{f_{ij}^{e}}. \end{array}$$

In the formula, *r* is the number of rows in the contingency Table; *c* is the number of columns in the contingency Table; *f*_*ij*_^0^ is the observed frequency; *f*_*ij*_^*e*^ is the expected frequency.

The formula for calculating the expected frequency of *f*^*e*^ is as follows.

(2) $$\begin{array}{c} f^{e}=\frac{RT}{n}*\frac{CT}{n}*n=\frac{RT*CT}{n}. \end{array}$$

In the formula, RT is the sum of the observation frequency of the row; CT is the sum of the observation frequency of the column.

By deriving the X^2^ statistic from the above formula, it can be seen that if the expected frequency and the observed frequency are the same, the X^2^ statistic is the smallest, which is 0, it can be inferred that these two variables are completely independent and have no correlation. If the difference between the expected frequency and the observed frequency is larger, the obtained X^2^ statistic is larger and the degree of correlation is higher [14].

## 4. Analysis of Results

### 4.1. Biopsy or Postoperative Pathology Results

The results of biopsy or postoperative pathological examination showed that 88 lesions were detected in 82 patients with liver nodular lesions, including 51 patients with benign lesions and 54 lesions, and 31 patients with malignant lesions, with 34 lesions. The nature of liver nodular lesions is shown in Table 1.

### 4.2. The Diagnostic Value of CEUS in Liver Nodular Lesions

Taking biopsy or pathological examination results as the gold standard, the four-table analysis CEUS has a sensitivity of 79.63%, a specificity of 82.35%, an accuracy of 80.68%, and a Kappa value of 0.603 in diagnosing benign and malignant liver nodular lesions, as shown in Table 2 and Figure 2.

### 4.3. Diagnosis of Liver Nodular Lesions by fMRI

Taking biopsy or pathological examination results as the gold standard, the four-table analysis of fMRI has a sensitivity of 83.33%, a specificity of 85.29%, an accuracy of 84.09%, and a Kappa value of 0.672 for the diagnosis of nodular benign and malignant liver lesions, as shown in Table 3 and Figure 3.

### 4.4. CEUS Combined with fMRI in the Diagnosis of Liver Nodular Lesions

1. A positive diagnosis by CEUS or fMRI is a positive result of the combined diagnosis, and a biopsy or pathological examination result is the gold standard, the four-table analysis of CEUS combined with fMRI in the diagnosis of nodular benign and malignant lesions of the liver is shown in Table 4.
2. Among the 54 benign lesions and 34 malignant lesions in the pathological examination results, the sensitivity of CEUS combined with fMRI in diagnosing benign and malignant liver nodule lesions was 94.44%, the specificity was 91.18%, and the accuracy was 93.18%, the Kappa value was 0.856, which was better than the single detection of the two, the accuracy of CEUS combined with fMRI diagnosis was statistically significant compared with CEUS and fMRI single detection (*χ*^2^  = 5.683, *P* < 0.055), as shown in Table 5.

## 5. Discussion

HCC is the most common primary malignant tumor of the liver and the second leading cause of human death. China is one of the countries with a high incidence of HCC, and its fatality rate ranks second in the cause of death from malignant tumors in my country, which seriously threatens human health. Some studies have found that most HCCs develop from atypical hyperplastic nodules, chronic liver inflammation is associated with various stages of hepatic parenchymal fibrosis, especially with end-stage liver disease (cirrhosis), and is the main cause of HCC. Therefore, the early noninvasive diagnosis and identification of liver nodular lesions are of great significance to improve the survival rate and prognosis of patients. Recent pathological, molecular biology and imaging studies suggest that the development of cirrhotic nodules to HCC is a multi-step cancerous process, including cirrhotic regenerative nodules, low-grade dysplastic nodules, and high-grade dysplastic nodules. A series of procedures and HCC. Currently, a pathological biopsy is still the gold standard for early clinical differential diagnosis of liver nodular lesions, but its application is limited due to its invasiveness. CT has a high diagnostic value for liver nodular lesions, but CT requires a large amount of contrast agents, the two contrast agents have nephrotoxicity and can cause many adverse reactions, so it is very important to find an accurate, error-free, and easy-to-operate differential diagnosis method [15]. 70%–75% of the blood supply to the liver is supplied by the hepatic artery, and 25%–30% is supplied by the portal vein, the process of the transformation from cirrhotic nodules to liver cancer is the process of capillary vascularization and angiogenesis in cirrhotic nodules, that is, the blood supply of the nodule changes from the main blood supply of the portal vein to the main blood supply of the hepatic artery. Therefore, the detection of liver nodular lesions is closely related to its blood supply, different nodular lesions in the liver have different enhancement methods, and different enhancement methods play a decisive role in the detection of lesions at different stages [16]. Compared with CT, CEUS can not only evaluate the nodular morphology of the liver but also clearly observe the blood flow of the hepatic artery, portal vein, and liver parenchyma after the contrast agent is immersed in the liver, which is specific for the diagnosis of liver nodular lesions. Studies have reported that the accuracy rates of CEUS in diagnosing cirrhotic nodules, dysplastic nodules, and HCC are 93.3%, 78.9%, and 85.5%, respectively. CEUS perfusion phase analysis can objectively reflect cirrhotic nodules and dysplastic nodules in the liver, as well as different perfusion patterns of micro-HCC, regular monitoring of cirrhotic nodules with CEUS, can prompt early warning and early diagnosis of micro-HCC, and improve the prognosis of patients [17]. The authors collected imaging data of 82 patients with liver nodular lesions and found that CEUS has a sensitivity of 79.63%, a specificity of 82.35%, an accuracy of 80.68%, and a Kappa value of 0.603 for the diagnosis of nodular benign lesions of the liver, among them, 2 cases of metastatic cancer may be due to increased blood vessels in cancer, this led to the misdiagnosis of hemangioma such as portal vein concentric enhancement, suggesting that CEUS can be used for the early differential diagnosis of liver nodular lesions, but the sensitivity is not good, and there is a certain missed diagnosis rate. MRI technology has high resolution and rapid image acquisition, and is currently widely used in clinical practice. fMRI is an emerging neuroimaging method, which is mainly used in the study of human and animal brain or spinal cord, recently, it has gradually become the main method for clinical diagnosis of liver diseases. Some studies have reported that MRI and fMRI can clearly show the changes in the shape and size of the harness in the state of liver disease, which is of great reference value for evaluating the diagnosis of chronic liver disease and the functional reserve of the liver. The results of this study found that the sensitivity of fMRI in diagnosing benign nodular liver lesions was 83.33%, the specificity was 85.29%, the accuracy was 84.09%, and the Kappa value was 0.672, suggesting that fMRI has a certain reference value in the differential diagnosis of benign and malignant liver sarcoidosis [18]. CEUS detected 43 lesions and fMRI detected 45 lesions, and the sensitivity was higher than that of CEUS, it can be seen that fMRI can make up for the deficiency of CEUS. Therefore, the authors' combined detection of the two with a sensitivity of 94.44%, a specificity of 91.18%, an accuracy of 93.18%, and a Kappa value of 0.856, which were both better than single detection, the reinforcement method is basically the same [19]. However, due to the difference in imaging methods between the two, the detection rate and differential diagnosis accuracy of liver nodular lesions are different, suggesting that CEUS combined with fMRI examination and biopsy or pathological methods are more consistent in diagnosing benign and malignant liver nodular lesions, its application may have a higher value in the early differential diagnosis of clinical liver nodular lesions, and can significantly improve its sensitivity and accuracy.

## 6. Conclusion

CEUS and fMRI have certain differential diagnosis values for the nature of liver nodular lesions, the combination of the two can improve the sensitivity and accuracy, and has more clinical application value; however, due to the small number of cases included in this study, there are certain deficiencies, and it is necessary to increase the sample size to further explore the diagnostic value of CEUS and fMRI for liver nodular lesions.

## Figures and Tables

**Figure 1:** NMR technique.

**Figure 2:** CEUS diagnosis of benign and malignant liver nodular lesions.

**Figure 3:** The results of fMRI diagnosis of nodular benign and malignant liver lesions.

**Table 1:** Biopsy or postoperative pathological findings.

Cases and lesions	Benign lesions						Malignant lesions			
	Hemangioma	Regenerative nodules	Focal fatty nodules	Focal fatty infiltration	Localized nodular hyperplasia	Total	Metastatic cancer	Hepatocellular carcinoma	Primary small liver cancer	Total
Number of cases (cases)	23	5	17	2	4	51	14	5	12	31

The number of lesions (pieces)	25	5	17	3	4	54	17	5	12	34

**Table 2:** CEUS diagnosis of liver nodular lesions (each).

CEUS	Biopsy or pathology		
	Benign lesions	Malignant lesions	Total
Benign lesions	43	6	49
Malignant lesions	11	28	39
Total	54	34	88

**Table 3:** Diagnosis of liver nodular lesions by fMRI (each).

fMRI	Biopsy or pathology		
	Benign lesions	Malignant lesions	Total
Benign lesions	45	5	50
Malignant lesions	9	29	38
Total	54	34	88

**Table 4:** Diagnosis of liver nodular lesions by CEUS combined with fMRI (each).

CEUS combined with fMRI	Biopsy or pathology		
	Benign lesions	Malignant lesions	Total
Benign lesions	51	3	54
Malignant lesions	3	31	34
Total	54	34	88

**Table 5:** Comparison of the diagnostic results of CEUS and fMRI alone and in combination for nodular benign and malignant liver lesions (%).

Detect	Sensitivity	Specificity	Accuracy
CEUS	79.63	82.35	80.68
fMRI	83.33	85.29	84.09
CEUS combined with fMRI	94.44	91.18	93.18
X^2^ value	4.853	1.107	5.683
*P* Value	0.028	0.293	0.017

## Data Availability

The data used to support the findings of this study are available from the corresponding author upon request.
